The article "Interventionally implanted port catheter systems for hepatic arterial infusion of chemotherapy in patients with primary liver cancer: A phase II-study (NCT00356161)" was published in 2013. Journal: BMC Gastroenterol.

# Interventionally implanted port catheter systems for hepatic arterial infusion of chemotherapy in patients with primary liver cancer: A phase II-study (NCT00356161)

**DOI:** 10.1186/1471-230X-13-125

**Published:** 2013-08-09

**Authors:** Marianne Sinn, Annett Nicolaou, Jens Ricke, Pjotr Podrabsky, Daniel Seehofer, Bernhard Gebauer, Maciej Pech, Peter Neuhaus, Bernd Dörken, Hanno Riess, Bert Hildebrandt

**Affiliations:** 1 CharitéCentrum für Tumormedizin, Medizinische Klinik mit Schwerpunkt Hämatologie, Onkologie und Tumorimmunologie, Campus Virchow Klinikum, Charité-Universitätsmedizin Berlin, Augustenburger Platz 1, D-13344 Berlin, Germany; 2 CharitéCentrum für Tumormedizin, Klinik für Strahlenheilkunde, Campus Virchow Klinikum, Charité-Universitätsmedizin Berlin, Augustenburger Platz 1, D-13344 Berlin, Germany; 3 Klinik für Radiologie und Nuklearmedizin, Otto-von-Guericke-Universität Magdeburg, Leipziger Str. 44, D-30120 Magdeburg, Germany; 4 CharitéCentrum für Chirurgische Medizin, Klinik für Allgemein-, Viszeral- und Transplantationschirurgie, Campus Virchow Klinikum, Charité Universitätsmedizin Berlin, Augustenburger Platz 1, D-13344 Berlin, Germany

**Keywords:** Hepatic arterial infusion, Infusions, Intra-arterial, Liver neoplasms, Hepatocellular cancer, Biliary tract cancer, Cholangiocellular carcinoma, Natriumfolinate, 5-fluorouracil, Oxaliplatin

## Abstract

**Background:**

Hepatic arterial infusion (HAI) of chemotherapy requires the implantation of a transcatheter application system which is traditionally performed by surgery. This procedure, but particularly the adjacent drug application via pump or port is often hampered by specific complications and device failure. Interventionally implanted port catheter systems (IIPCS) facilitate the commencement of HAI without need for laparatomy, and are associated with favorable complication rates. We here present an evaluation of the most important technical endpoints associated with the use of IIPCS for HAI in patients with primary liver cancers.

**Methods:**

70 patients (pts) with hepatocellular (HCC, n=33) and biliary tract cancer (BTC, n=37) were enrolled into a phase II –study. Of those, n=43 had recurrent disease and n=31 suffered from liver-predominant UICC-stage IVb. All pts were provided with IIPCSs before being treated with biweekly, intraarterial chemotherapy (oxaliplatin, 5-Flourouracil, folinic acid). The primary objective of the trial was defined as evaluation of device-related complications and port duration.

**Results:**

Implantation of port catheters was successful in all patients. Mean treatment duration was 5.8 months, and median duration of port patency was not reached. Disease-progression was the most common reason for treatment discontinuation (44 pts., 63%), followed by chemotherapy-related toxicity (12 pts., 17%), and irreversible device failure (5 pts., 7%). A total of 28 port complications occurred in 21 pts (30%). No unexpected complications were observed.

The article "Interventionally implanted port catheter systems for hepatic arterial infusion of chemotherapy in patients with primary liver cancer: A phase II-study (NCT00356161)" was published in 2013. Journal: BMC Gastroenterol.

**Conclusions:**

HAI via interventionally implanted port catheters can be safely applied to patients with primary liver tumors far advanced or/and pretreated.

## Background

Hepatocellular carcinoma (HCC) and biliary tract cancer (BTC) represent the most common primary liver malignancies, with steadily increasing incidences in Europe and North America. At first glance, tumors arising from the liver parenchyma and those developing from the biliary tract exhibit a number of dissimilarities, such as differences with regard to incidence and risk factors. However, both cancers also share a number of features that allow a combined consideration [1-3].

Surgery and - in small HCCs - orthopic liver transplantation represent potentially curative treatment options, but the majority of patients with HCC and BTC are diagnosed in advanced disease stages. For irresectable patients, the prognosis is dismal on principle, although recent studies on medical treatment revealed substantial progress for both cancer types [4,5]. Despite those encouraging results, median survival rates in the respective trials - where only patients with advanced disease were included - did not exceed 12 months [6,7] so that further improvements in the treatment of patients with advanced BTC and HCC are worthwhile.

One possible explanation for the discouraging results of chemotherapy in advanced liver cancers may be that the systemic drug concentrations achieved are not efficient enough to warrant loco-regional tumor control. Indeed, both BTC and HCC typically remain restricted to the liver or, at least, liver-predominant even in advanced disease stages. From a theoretical point of view, regional chemotherapy approaches may be considered more effective than systemic drug application in most of those patients [8,9].

Valid data on this matter are restricted to the application of transarterial chemoembolisation (TACE) in patients with intermediate stage HCC-patients. TACE can be regarded as current standard for the treatment of HCC-patients with irresectable, but localized multinodular HCC with maintained liver function (BCLC group B) where it yields overall survival rates in the range of 20 months [8,10,11]. The observation that TACE achieves better results than transarterial embolization alone [12] supports the hypothesis that the application of regional chemotherapy relevantly contributes to the overall efficacy of the approach. Data on the use of drug eluting beeds (DEB) for TACE further suggest that delayed release of chemotherapeutic agents in the scope of this approach results in elevated regional drug concentration [13,14]. As those are in turn considered causal for the superior clinical results achieved, one may reason that the efficacy of chemotherapy application in the scope of TACE is dose-dependent.

The article "Interventionally implanted port catheter systems for hepatic arterial infusion of chemotherapy in patients with primary liver cancer: A phase II-study (NCT00356161)" was published in 2013. Journal: BMC Gastroenterol.

Most patients with advanced BTC or HCC suffer from severe restriction of liver function and concomitant disease. Therefore, they are not eligible for a combined treatment with tumor embolisation and regional chemotherapy. Taking the above-mentioned dose-dependency of regional drug application in the scope of TACE as basis, one strategy to further improve the outcome of patients with advanced liver-limited or –predominant BTC and HCC may be the use of modern regional chemotherapy approaches in the scope of hepatic arterial infusion (HAI) [15,16].

HAI of chemotherapy enables repetitive delivery of high intrahepatic drug concentrations in the absence of synchronous embolisation of liver vasculature with acceptable toxicity. Extensive experience with the technique has been gained in patients with isolated liver metastases of colorectal cancer (CRC). A number of randomized trials on HAI using FUDR or 5-FU in patients with irresectable colorectal liver metastases or after liver resection have been performed since the 1980ies, but achieved inconsistent results. Besides inadequate study designs (particularly in the older trials) technical problems with the application devices employed appear as major reasons why the method failed to become a standard treatment outside of clinical trials [17-19].

During the past decade, the feasibility of HAI was relevantly improved by the introduction of interventionally implanted port catheter systems (IIPCS). IIPCS enable initiation of HAI without laparatomy, and are associated with favourable complication and failure rates [20-22]. Most experiences with the technique have again been gained in patients with colorectal liver metastases [22], and it has not been thoroughly investigated in patients with primary liver cancers so far.

In order to further define practicability and safety of our HAI-approach applied via IIPCS we included patients with advanced HCC and BTC in a phase 2-trial in which technical endpoints (complication rates, safety of device and regional therapy) were defined as primary objectives. The intraarterial chemotherapy schedule consisting of oxaliplatin, folinic acid, and 5-flourouracil (OFF) was firstly evaluated in patients with colorectal liver metastases. As 5-FU or its oral prodrug capecitabine combined with Oxaliplatin are drugs considered particularly effective in patients with advanced BTC [23,24], we wanted to evaluate the efficacy and safety of HAI with oxaliplatin and 5-fluorouracil/folinic acid (OFF) in patients with liver predominant disease. For HCC, more recent data showed efficacy for the intraarterial application via HAI if 5-FU alone or in combination with the platinum-derivate cisplatin [16,25].

The article "Interventionally implanted port catheter systems for hepatic arterial infusion of chemotherapy in patients with primary liver cancer: A phase II-study (NCT00356161)" was published in 2013. Journal: BMC Gastroenterol.

Herein, we report our experience with the regional OFF regimen via HAI in a larger cohort of patients with advanced, irresectable BTC/HCC, focusing our presentation on the primary study objectives “complication rates” and “safety of device and regional therapy”.

## Methods

### Study design, patients´ collective and eligibility criteria

Patients with primary liver cancer were prospectively enrolled into a phase II-study on the evaluation of technical complications associated with the use of interventionally implanted port catheter systems (IIPCS) in patients with cancers confined to the liver between 2004 and 2010 (ClinicalTrials.gov Identifier: NCT00356161). The protocol was approved by the local ethics committee (EC of the Charité University Clinic, Berlin, Germany), and a detailed written informed consent was obtained from every patient prior to treatment.

Adult patients were eligible if they had histologically proven, irresectable, primary or recurrent hepatocellular cancer (HCC) or intracellular cholangiocarcinoma (ICC), an ECOG performance status of 0–2, an estimated life expectancy of ≥ 3 months, and no contraindication against the initiation of hepatic arterial infusion of chemotherapy. Main exclusion criteria were evident extrahepatic manifestations (abdominal lymph nodes > 25 mm, pulmonary lesions > 15 mm), severe alteration of liver function (cirrhosis, prothrombin time<50%), active viral hepatitis, portal vein thrombosis, previous liver irradiation, impaired coagulation, significant concomitant disease, history of second malignancy. Previous chemotherapy was no exclusion criterion for this study.

Primary objective was the evaluation of technical endpoints associated with the use of IIPCS for the application of HAI, comprising complications associated with port implantation and adjacent regional chemotherapy, port duration (defined as time to port occlusion), and reasons for primary and secondary device failure. Secondary endpoints included the evaluation of a standardized approach of chemotherapy application according to the different treatment indications, chemotherapy toxicity, response and survival rates. This report refers to the evaluation of the primary endpoint of the study for the subgroup of patients with primary liver cancer (e.g. hepatocellular and intrahepatic cholangiocellular cancer).

The article "Interventionally implanted port catheter systems for hepatic arterial infusion of chemotherapy in patients with primary liver cancer: A phase II-study (NCT00356161)" was published in 2013. Journal: BMC Gastroenterol.

The port implantation procedure was performed as previously described in detail by Ricke et al. ([21]). A standard angiography catheter was placed in the hepatic artery and subcutaneously connected to a port system (Titakath; Innovent, Hürth, Germany) inferior to the groin, using a titanium connector (Arrow, Reading, PA, USA). Functionality of the system was examined by digital subtraction angiography (DSA), and by requirement complemented by a scintigraphy using (99m)Tc-labelled macroaggregated albumin. If significant extrahepatic perfusion was detected after primary successful implantation of the IIPCS, treatment was interrupted. The device was revised if this appeared promising from the view of the interventional radiologist and the patient had responded to treatment. DSA was repeated before each treatment course.

### Interventions

#### Hepatic arterial infusion of chemotherapy

Patients with primary liver cancer received a biweekly combination therapy of intraarterial oxaliplatin (85 mg/m^2^, diluted in 50 ml glucose 5%, 120 minutes), followed by an intraarterial mixture of natriumfolinate (170 mg/m^2^) and 5-FU (600 mg/m^2^, both diluted in 50–100 ml saline, 120 minutes; regional “OFF”-schedule). For 5-FU, a dose-escalation of 10% per cycle was performed until the occurrence of adverse reactions (WHO I-II). Supportive treatment consisted of a standard antiemetic regimen (Dexamethasone, HT3-Antagonist). The port system was flushed with 10 ml glucose 5% after the application of oxaliplatin, and blocked with either 5000 units unfractionated heparine or 3000 anti-Xa units Nadroparine diluted in 5 ml of saline after every application. Data on the feasibility and toxicity of the regional chemotherapy schedule has been previously published in [21,22].

### Evaluations

#### Pretreatment evaluation and follow-up

Each patients´ history was recorded, and clinical examination and routine laboratory status were performed within the 14 days preceeding the first chemotherapy application. Basic imaging consisted of an abdominal CT or MRT and chest-X-ray or CT. Clinical evaluation, a full blood count and clinical chemistry were repeated before every HAI-application. Assessment of toxicity was performed according to WHO-criteria.

Response evaluation was performed according to WHO criteria and repeated in 3-monthly intervals. After the end of treatment, patients were seen at least every 3 months. Follow-up consisted of clinical visits, laboratory and imaging until disease progression, initiation of salvage treatment or death. The efficacy analyses included objective response rates, as well as, progression free- and overall survival.

The article "Interventionally implanted port catheter systems for hepatic arterial infusion of chemotherapy in patients with primary liver cancer: A phase II-study (NCT00356161)" was published in 2013. Journal: BMC Gastroenterol.

Treatment was interrupted in case of irreversible loss of port function, WHO toxicity of grade IV (except for haematotoxicity), or disease progression after escalation of treatment. The drug dosages were reduced if WHO-toxicity III° or haematotoxicity III/IV° appeared in between of two treatment courses, or if toxicity >WHO I° was ongoing on the first day of the following cycle (except for leukopenia: >WHO II° and thrombopenia: >II°). For combination regimens, it was at the physicians discretion to reduce the dose of all compounds or only of one drug.

#### Port complications, port duration, and toxicity

Port-related adverse events were assessed from the date of successful implantation. Patency and integrity of the port system was documented by DSA, complemented by a scintigraphy of the liver with Tc-99m labeled macroaggregated albumine if gross pathological findings were observed. Port duration was defined as functional device with or without revision, but without requirement for explantation of the entire system. Patients in which HAI was stopped because of disease progression were censored at the last application of HAI.

#### Statistical evaluations

Differences between proportions were analyzed by using chi-square tests. Mann–Whitney tests were employed to compare quantitative and ordinal variables. The univariate analyses of port duration were calculated according to the Kaplan-Meier method, and comparisons between groups were calculated by using Log-Rank tests. A two-sided p-value less than 0.05 was considered to prove significance for all tests performed. All analyses were performed by using the SPSS 18.0 software package.

## Results

### Patients’ characteristics, treatment characteristics, and efficacy

Between 2004 and 2010, a total of 70 pts with primary liver cancers were enrolled (n=33 HCC, n=37 ICC). Most patients had recurrent disease and were pretreated by resection, chemotherapy, interventional procedures, or more than one of those modalities. Five patients with HCC had previously undergone orthopic liver transplantation (Table 1).

**Table 1:** Patients’ characteristics

**Characteristics**	**n (Total n=70)**	
	**HCC *(n=33)***	**ICC *(n=37)***
Age (median/range)	66 (38–76)	59 (41–79)
Gender (f/m)	8/25	22/15
Primary tumour:		
Primary/recurrent	8/25	19/18
Grading (G1/G2/G3/n.a.)	1/11/20/12	3/17/7/10
Child-Pugh class A/B/C/n.a.	25/3/1/4	--
Stage IVb	10	21
Pretreatment:		
Hepatic resection	18	12
Liver transplantation	5	0
Sorafenib/Chemotherapy	1	6
Chemoembolisation	12	1
Local ablation (RFA, brachytherapy)	2	2
Elevated AFP/Ca 19-9	24	32

Port implantation was successful and regional therapy was initialized in all patients, e.g. no case of primary port failure occurred. Disease progression was the most common reason for treatment termination (n=44), followed by chemotherapy-toxicity as second leading cause (n=12). Only a minority of patients (n=5) had to stop HAI due to irreversible port dysfunction. There number of device-related complications was acceptable (28 episodes in 21 patients), revisions of the device were required in 15 patients (Table 2).

The article "Interventionally implanted port catheter systems for hepatic arterial infusion of chemotherapy in patients with primary liver cancer: A phase II-study (NCT00356161)" was published in 2013. Journal: BMC Gastroenterol.

**Table 2:** Treatment characteristics

**Number of patients**	**70**
**Number of treatment cycles**	**562**
Range	1-34
Mean	8
**Reason for termination of HAI**	
Disease progression (intrahepatic n=11, extrahepatic n=16, both n=17)	44 (63%)
Chemotherapy-related toxicity	12 (17%)
Port complication	5 (7%)
Post-progression HAI	4 (6%)
Refusal	4 (6%)
Loss of follow up	1 (1%)
**Port complications per patient**	
≥1 complication	21 (30%)
≥3 complications	3 (4%)
≥ 1 revision	15 (21%)

Port-related complications mostly consisted of vascular events, typically subtotal thrombosis of the hepatic artery or one of its branches, or dislocation of the catheter tip. Non-vascular problems were less frequent, but infections of the port chamber accounted for most of the treatment-limiting port-complications (Table 3a and b). In one patient, disease progression after intraarterial chemotherapy was associated with deterioration of portal hypertension and, consecutively, fatal gastrointestinal haemorrhage. This patient had undergone revision of his IIPCS due to dislocation of the catheter tip and infection of the port chamber two days before.

**Table 3:** Port complications

***a) Overall complications***			
		***Abs.***	***%***
**Number of complications**		**28**	**100**
***vascular***		**17**	**61**
	Dislocation of catheter tip	7	25
	Thrombosis	8	29
	Reflux	2	7
***non vascular***		**11**	**39**
	Leakage	2	7
	Infection of port chamber	7	25
	others	2	7
***b) Treatment -limiting complications***			
		***Abs.***	***%***
**Number of complications**		**5**	**100**
***vascular***			
	Thrombosis	1	20
***non vascular***			
	Infection	4	80

Patient received a median of 6 chemotherapy applications. Median treatment duration was 3.9 months. Median duration was of port patency was not reached. Rates of patients with functional devices at 12 months were 13% (Figure 1). Median time to progression was 5.8 months, and overall survival was 9.0 months.

**Figure 1:** Kaplan-Meier estimation of cumulative port patency.

#### Chemotherapy toxicity

A total of 41 WHO grade 3/4 adverse events (AEs) were recorded regardless of their causality to treatment and occurred in 30 patients (43%) as follows: Infection n=15, abdominal pain or bleeding n=7, diarrhoe n=6, haematological n=5, polyneuropathy n=1, others n=7. In 12 patients (17%) severe AEs were causally related to chemotherapy and thus resulted in treatment interruption (Table 2).

The article "Interventionally implanted port catheter systems for hepatic arterial infusion of chemotherapy in patients with primary liver cancer: A phase II-study (NCT00356161)" was published in 2013. Journal: BMC Gastroenterol.

## Discussion

The study collective evaluated herein consists of a heterogenous group of 70 patients suffering from hepatocellular or intrahepatic cholangiocellular cancer with liver-limited or liver-predominant disease. For most of them no established treatment option was available. Patients were provided with an IIPCS and adjacent HAI using oxaliplatin, folinic acid, and 5-FU (regional “OFF”-schedule) in the scope of a study that was intentionally designed for technical endpoints in order to get a more detailed insight into the practicability of the approach. Thus we were able to give a detailed description on the technical aspect of HAI applied via IIPCS in primary liver cancer for the first time. Results obtained in the first phase of this research program referred to the treatment of patients with colorectal liver metastases and have already been reported [22].

It was found that implantation of IIPCS was feasible in all patients, and that the rate of device related-complications was relatively low. In addition, the proportion of patients with treatment discontinuation due to port-failure compares favourably to our previously reported experience in colorectal liver metastases, and the same holds true for the Kaplan-Meier estimation of overall port patency [22,26]. In the interpretion of these results one has to consider the short average treatment duration. Indeed, when calculating overall port patency as given in Figure 1, as much as 21 patients were censored within the first 6 months of treatment, and the rate of devices functioning at 12 months was only 13%. This clearly reflects that disease progression preceded port failure in the majority of patients. However, our findings on progression-free and overall survival may suggest a certain activity of regional chemotherapy that will be further analysed and reported in a separate publication.

Another finding of importance may be our observation that the high proportion of patients suffering from pre-treated and far advanced tumours did not seriously counteract successful port implantation and regional chemotherapy. Even though we and others already demonstrated that HAI administered via IIPCS is feasible and at least non-inferior when compared with surgically implanted systems in a nonrandomised fashion [22,27,28], these data refer to patients with colorectal liver metastases - and thus to an entity which is usually characterised by the absence of primary liver disease. Thereby, our results support the hypothesis that HAI via IIPCS can be also applied to patients with liver neoplasms suffering from recurrent disease, high tumour burden, and/or cirrhosis.

The article "Interventionally implanted port catheter systems for hepatic arterial infusion of chemotherapy in patients with primary liver cancer: A phase II-study (NCT00356161)" was published in 2013. Journal: BMC Gastroenterol.

We observed grade 3 and 4 adverse events in 43% of patients enrolled, and treatment interruptions due to grade 3 and 4 toxicity were required in 17% of patients. In the pivotal studies on sorafenib in HCC [7] grade 3 or 4 toxicity per patient was reported in 54% (placebo arm) and 52% (sorafenib arm) of patients treated. The respective percentages for cisplatin/gemcitabine [25] were 69 (gemcitabine) and 71 (gemcitabine/cisplatin). It seems that a high proportion of patients with advanced liver cancers (e.g. 54% in the placebo arm of the HCC-trial) will become symptomatic without treatment in a considerable short period of time, and that the application of standard chemotherapy does not relevantly improve this rate. In the light of those data our rates of severe adverse events appear acceptable.

Discussing our finding in the context of the literature, we already mentioned in the introduction that most data available on the use of transcatheter techniques in primary liver neoplasms so far refer to the application of transarterial chemoembolisation (TACE) [29-32]. The few disease-specific trials on HCC-patients treated by hepatic arterial infusion without synchronous use of embolising agents employed repetitive catheterisation techniques [25] or IIPCS [33]. In the latter, HAI using 5-FU and cisplatin was administered to 52 patients with advanced HCC, and one failure of the IIPCS was reported that was caused by thrombosis of the hepatic artery. The experience on HAI in patients with BTC is also limited, although first studies already date back to the 1980ies [34]. One recent series on 11 patients treated with HAI via IIPCS did not explicitly state on the device-related complications observed, whereas irreversible dysfunction was reported in 5 out of 16 patients in another one [35,36]. Two further trials in which patients with both HCC and ICC were included and treated with HAI applied via surgically implanted pumps have recently reported by the workgroup of the Memorial Sloan Kettering Cancer Center [15,37]. Postoperative complications were observed in 8 out of 34 (23,5%) in the first, and in 4 out of 56 (7,1%) in the second of these studies.

To sum it up, the experience with the use of HAI in primary liver neoplasms is still very limited and is still far removed from representing an established treatment option. Data available did not report on excess technical problems so that our results support the assumption that that the use of IIPCS is practicable and safe in patients with advanced liver neoplasms. But even if progress of minimally-invasive techniques has considerably simplified the application of intraarterial transcatheter therapies during the past decade, this is not reflected by a higher number of clinical trials published on HAI for any indication. In colorectal liver metastases – the main field of HAI-application in the 5-FU-era – a rapid progress in drug development took place during the past 15 years, and studies on HAI did not manage to keep up with this. In HCC and BTC, recent studies on systemic drug therapy produced the first considerable progress in medical treatment for these neoplasms for the past 30 years, but there remains a substantial need for the improvement of treatment results.

The article "Interventionally implanted port catheter systems for hepatic arterial infusion of chemotherapy in patients with primary liver cancer: A phase II-study (NCT00356161)" was published in 2013. Journal: BMC Gastroenterol.

Hepatic arterial infusion in patients with primary liver neoplasm has a striking rationale, because it enables the application of high drug concentrations without corresponding increase in overall toxicity. The introduction of interventionally implanted application systems largely facilitated the initiation of regional chemotherapy. Our results support the hypothesis that HAI via IIPCS is safe, and requires further evaluation in patients with primary liver cancers.

## Conclusions

Hepatic arterial infusion via interventionally implanted port catheters can be safely administered to a prospective collective of patients with liver tumors, including a high proportion of patients with recurrence, high tumor burden and/or cirrhoses.

## Competing interests

*Bert Hildebrandt* has received honoriaria (below 10000 Euro each) from Roche, Sanofi-Avantis and Merck, and research funding from Sanofi-Aventis (10–99000 Euro). Parts of t he manuscript were presented at the annual meeting of the Deutsche Gesellschaft für Hämatologie und Onkologie (DGHO) in 2010.

## Authors’ contributions

MS: contributed to provision of patients, collection and assembly of data, data analysis and interpretation, and manuscript writing. AN: contributed to provision of patients, collection and assembly of data, data analysis and interpretation, and manuscript writing. JR was involved into the conception and design of the study, provision of patients, collection and assembly of data, data analysis and interpretation, and manuscript writing. He introduced and performed the interventional implantation of hepatic arterial port catheters. PP was involved into the provision of patients, and interventional implantation of hepatic arterial port catheters. DS: was involved into the provision of patients, collection and assembly of data. MP: was involved into the design of the study, provision of patients, and interventional implantation of hepatic arterial port catheters. BG: was involved into the provision of patients and interventional implantation of hepatic arterial port catheters. PN contributed to the conception and design of the study and provision of patients, and gave administrative support. BD contributed to the conception and design of the study and gave administrative support. HR contributed to the conception and design of the study, as well as, to the provision of patients. He prescribed and administered regional chemotherapy. He gave administrative support and was involved into manuscript writing. BH contributed to the conception and design of the study, provision of patients, collection and assembly of data, data analysis and interpretation. He prescribed and administered regional chemotherapy. He has written the first draft of the manuscript and implemented the revisions of the co-authors. All authors have revised the manuscript critically, and have given final approval of the version to be published.

The article "Interventionally implanted port catheter systems for hepatic arterial infusion of chemotherapy in patients with primary liver cancer: A phase II-study (NCT00356161)" was published in 2013. Journal: BMC Gastroenterol.

## Pre-publication history

The pre-publication history for this paper can be accessed here:

http://www.biomedcentral.com/1471-230X/13/125/prepub
